This article has been retracted.

# Mendelian Randomization Study of Causal Relationship between Omega-3 Fatty Acids and Risk of Lung Cancer

**DOI:** 10.1155/2022/2786567

**Published:** 2022-05-31

**Authors:** Xin Liu, Yanzhi Peng, Ru Tao, Ling Meng, Xuehua Li

**Affiliations:** ^1^Department of Respiratory and Critical Care Medicine, The Second Affiliated Hospital of Shandong First Medical University, Tai'an, 271000 Shandong, China; ^2^Medical Oncology, Feicheng Hospital Affiliated to Shandong First Medical University, Feicheng, 271600 Shandong, China; ^3^School of Nursing, Shandong First Medical University, Tai'an, 271000 Shandong, China; ^4^Department of Respiratory Medicine, The Second Affiliated Hospital of Shandong First Medical University, Tai'an, 271000 Shandong, China

## Abstract

**Objective:**

Evidence suggests that omega-3 fatty acid intake exerts a protective effect on lung cancer, but its causal association with risk of lung cancer remains uncertain. This study attempts to clarify the causal effect of omega-3 fatty acids on lung cancer utilizing genome-wide association study (GWAS) data with Mendelian randomization (MR) approach.

**Methods:**

This study acquired omega-3 fatty acid data from the UK Biobank and data of lung cancer patients from the Consortium and International Lung Cancer Consortium (ILCCO). Single-nucleotide polymorphisms (SNPs) associated with omega-3 fatty acids were screened as instrumental variables (IVs) in line with the criteria of *p* < 5*E* − 8, linkage disequilibrium *R*^2^ > 0.001 and distance < 10000 kb. Through inverse variance weighted (IVW), MR-Egger, weighted median, simple mode, and weighted mode, causal association between omega-3 fatty acids and risk of lung cancer was evaluated. Cochran's *Q* test was applied for a heterogeneity test. The pleiotropy and horizontal pleiotropy among IVs were evaluated via MR-Egger regression intercept analysis.

**Results:**

Totally, 42 SNPs associated with omega-3 fatty acids were identified as IVs. According to the results of IVW (OR (95% CI): 0.899 (0.817, 0.990), *p* = 0.03), MR-Egger (OR (95% CI): 0.856 (0.750, 0.977), *p* = 0.026), weighted median (OR (95% CI): 0.899 (0.817, 0.990), *p* = 0.001), simple mode (OR (95% CI): 0.901 (-0.678, 1.199), *p* = 0.478), and weighted mode (OR (95% CI): 0.859 (0.782, 0.944), *p* = 0.003), omega-3 fatty acids showed a causal association with low risk of lung cancer. No genetic pleiotropy or horizontal pleiotropy was found according to MR-Egger regression intercept analysis.

**Conclusion:**

Our findings provide sufficient evidence that omega-3 fatty acids are causal protective factors of lung cancer. Despite this, further work is required for elucidating the potential mechanisms.

## 1. Introduction

Lung cancer represents the leading cause of cancer-related deaths globally, occupying 1.76 million death cases in 2018 [1]. Small-cell lung carcinoma (SCLC) and non-SCLC (NSCLC) are two major subtypes [2], which separately account for 15% and 85% of all lung cancer cases [3, 4]. The five-year survival of lung cancer remains approximately 19% because over 50% NSCLC cases are diagnosed as metastasis [5]. Early detection of lung cancer depends upon computed tomography (CT), and lung tissue biopsy can confirm CT-derived diagnosis, but it is of high invasiveness during surgery [6]. Hence, prevention especially dietary pattern remains the best way to deal with lung cancer [7].

Omega-3 fatty acids exert crucial effects on human health as well as various diseases, which contain *α*-linolenic acid (ALA), eicosapentaenoic acid (EPA), and docosahexaenoic acid (DHA) [8]. They can be acquired from ALA-containing plant oils; furthermore, EPA and DHA can be supplemented via eating fatty fishes [9]. Omega-3 fatty acids are the key components of many parts of the body [10, 11]. For instance, DHA is distributed in the cell membrane, while EPA and DHA are precursors of metabolites acting as lipid mediators and effective in prevention or treatment of a few diseases [12]. Experimental evidence supports the relationship between Omega-3 fatty acid intake and low risk of lung cancer. Specifically, Siena et al. reported that electrophilic derivatives of omega-3 fatty acids suppressed growth of lung cancer cells [13]. Moreover, omega-3 fatty acids mediated endoplasmic reticulum stress and ameliorated acquired gefitinib resistance for lung cancer [14]. Omega-3 fatty acids mediated the generation of inflammation-related molecules (known as eicosanoids) as well as inflammatory response [15]. Previous epidemiology and meta-analysis examined the putative relationship between omega-3 fatty acid consumption and lung cancer [16, 17]. Nevertheless, these studies cannot contain an overall assessment and incorporation of bias or uncertain factors for supporting causal relationships. In traditional observational epidemiology, exposure-outcome associations can be influenced by confounding factors and reverse causal associations, thereby limiting in causal inference [18, 19]. To fill this gap, we applied Mendelian randomization (MR) to evaluate the causal effect of omega-3 fatty acids on lung cancer on the basis of genome-wide association study (GWAS) data. MR approach employs single-nucleotide polymorphisms (SNPs) as instrumental variables (IVs) to infer causal associations between exposure and outcomes, which can overcome confounding factors and the influence of reverse causality association on causal inference [20, 21]. Our findings demonstrated that omega-3 fatty acids were causal protective factors of lung cancer.

## 2. Materials and Methods

### 2.1. Genome-Wide Association Study (GWAS) Summary Data

To ensure that the MR analysis had high power for estimating the causal effect and the reproducibility of our results, this study collected publicly available genetic summary data from two large consortiums (the UK Biobank [22] and the International Lung Cancer Consortium (ILCCO)). GWAS summary data on omega-3 fatty acids were accessed from the UK Biobank, containing 114,999 samples and 12,321,875 single-nucleotide polymorphisms (SNPs), as shown in Table 1. GWAS summary data on lung cancer were required from the ILCCO (http://ilcco.iarc.fr/), including 18,313 European lung cancer patients. Data of above patients were on the basis of GWAS of European cohorts: MDACC, ICR, NCI, and IARC. Summary data of 8,893,750 SNPs were also required from the ILCCO (Table 1).

### 2.2. SNPs Associated with Omega-3 Fatty Acids as Instrumental Variables (IVs)

The screening criteria of associated with omega-3 fatty acids were as follows: (1) *p* < 5*E* − 8 indicated a high correlation between SNPs and omega-3 fatty acids. (2) Linkage disequilibrium (LD) describes the correlation between genetic variants, usually caused by the proximity of physical locations between genetic variants. When LD exists between genetic variants, the information provided by each genetic variant is not independent, and when these nonindependent genetic variants are used as IVs, it will lead to biased effect estimates. Here, *R*^2^ > 0.001 indicated that SNPs were independent of each other to avoid the bias caused by LD that represented a nonrandom association of alleles at different loci. The SNPs associated with omega-3 fatty acids were used as IVs. (3) The distance between each other was <10000 kb. Thereafter, the data extracted from the two databases were consolidated, and the effect value of exposure and outcomes corresponded to the same effect allele. The information of each SNP was collected, including the main alleles, allele frequencies, *β* coefficients, *p* values, and standard errors (SEs).

### 2.3. Mendelian Randomization (MR) Analyses

Five MR analyses including inverse variance weighted (IVW), MR-Egger, weighted median, simple mode, and weighted mode were applied to estimate the association between omega-3 fatty acids and risk of lung cancer. IVW is the standard method for summarizing data in MR, which does not require individual-level data, and can directly use aggregated data to calculate causal effect sizes. Mean IVW estimates of SNP ratios were calculated by regression of the SNP-omega-3 fatty acid association with the SNP-lung cancer association. Median estimates include weighted median, simple mode, and weighted mode. Impact effects were estimated using the weighted median method, and the weighted empirical distribution function of the ratio estimates for all selected SNPs was calculated. The weighted median method allowed SNPs with stronger effects to contribute more to causal estimates and reduced bias in causal effect estimates when fewer SNPs were effective tools. MR-Egger analysis was performed, which assumed that horizontal variability was independent of SNP exposure effects (inside assumption), allowing for a nonzero intercept in regression and unbalanced horizontal variability for all SNPs. MR-Egger regression was a weighted linear regression of estimates of the effect of SNP-lung cancer risk and SNP-omega-3 fatty acids. MR-Egger could provide a valid causal effect assessment when all SNPs were ineffective tools. All results were expressed by odds ratio (OR) and its 95% confidence intervals (CI), and *p* < 0.05 was considered statistically significant. To visualize the results of statistical analysis and visualize the statistical effects of each SNP, the data analysis function of the MR-based platform was used to draw the forest plot and scatter plot of SNP-related omega-3 fatty acids and lung cancer risk.

### 2.4. Heterogeneity and Pleiotropy Test

MR analyses could have heterogeneity due to differences in platforms, experimental conditions, inclusion populations, and SNPs, thereby biasing estimates of causal effects. In our study, MR-Egger regression analysis was presented for assessing the underlying pleiotropic effects of SNPs as IVs. MR-Egger regression intercept is a useful indicator of directional horizontal pleiotropy drives the results from MR analyses [23]. IVW and MR-Egger regression analyses were utilized for detecting heterogeneity. The heterogeneity was quantified with Cochran's *Q* test. *p* < 0.05 indicated significant heterogeneity.

### 2.5. Statistical Analysis

All statistical analyses were implemented utilizing TwoSampleMR package (version 0.4.25) in R (version 3.6.2).

## 3. Results

### 3.1. Characteristics of SNPs Associated with Omega-3 Fatty Acids as IVs

In the UK Biobank, 42 SNPs (including rs10184054, rs10455872, rs11242109, rs112875651, rs1132899, rs11563251, rs1167998, rs11681659, rs117143374, rs117733303, rs12226389, rs1260326, rs13424225, rs139974673, rs143355652, rs1672811, rs174564, rs1800978, rs261290, rs3018731, rs34663616, rs35135293, rs4000713, rs58542926, rs6129624, rs62466318, rs629301, rs633695, rs6601924, rs6693447, rs673335, rs6882345, rs72789541, rs73109460, rs737338, rs77960347, rs7819706, rs7924036, rs7970695, rs9304381, rs964184, and rs9987289) were significantly associated with omega-3 fatty acids according to the criteria of *p* < 5*E* − 8, LD *R*^2^ > 0.001, and distance < 10000 kb, which were available in the ILCCO cohort. These SNPs were eligible for MR analyses. The details of the SNPs and the strength and magnitude of their correlations to omega-3 fatty acid and lung cancer are listed in Table 2. As illustrated in Figure 1, forest plot showed the estimates for each SNP on lung cancer.

### 3.2. Casual Effects of Omega-3 Fatty Acids on Risk of Lung Cancer

Figure 2 shows scatter plots of the SNP-lung cancer associations against the SNP-omega-3 fatty acid associations with five MR approaches, which visualized causal effect estimate for each individual SNP on lung cancer.  Table 3 shows causal effect estimates of omega-3 fatty acids on risk of lung cancer from five MR approaches. In the IVW MR analysis, the OR of lung cancer for omega-3 fatty acid intake was 0.899 (95% CI: 0.817-0.990; *p* = 0.03). Estimates were concordant and similar in size in the MR-Egger (OR (95% CI): 0.856 (0.750-0.977), *p* = 0.026), weighted median (OR (95% CI): 0.899 (0.817-0.990), *p* = 0.001), and weighted mode (OR (95% CI): 0.859 (0.782-0.944), *p* = 0.003) approaches, which supported a protective effect of omega-3 fatty acids on lung cancer. However, no statistical significance was found for simple mode approach.

### 3.3. Heterogeneity and Pleiotropy Test

Cochran's *Q* of IVM analysis showed that there was no heterogeneity among SNPs (*p* = 0.240). Moreover, MR-Egger regression analysis demonstrated that SNPs could have no-horizontal pleiotropy between omega-3 fatty acids and risk of lung cancer (*p* = 0.293; Table 3). Funnel plot showed that when using a single SNP as an IV, the point representative of the causal association effect was symmetric distribution, indicating that the cause was less likely to be affected by underlying bias (Figure 3).

## 4. Discussion

In MR studies, the effect relationship between exposure and outcome is not affected or distorted by confounders and reverse causal associations, which has unique advantages for causal inference of exposure factors [24]. The mature development of GWAS has laid the foundation for the development of MR research and also has opened a new door for the study of lung cancer risk [25]. This study adopted large-scale GWAS summary data to explore the causal relationship between omega-3 fatty acids and risk of lung cancer with MR approaches. SNP data of this study were all from the European cohorts, which avoided the bias caused by different populations. Nevertheless, the generalizability of our conclusion was uncertain due to the European cohort. Our MR analyses were based on the following assumptions: (1) SNPs were related to exposure factor-omega-3 fatty acids. This process was based on the GWAS research, and the appropriate SNPs were selected as IVs; (2) the formation of IVs was regarded as a process of random allocation, which was independent of confounding factors; (3) IVs can only affect the outcome-lung cancer through the exposure factor-omega-3 fatty acids. Our results demonstrated that there was a negative causal association between omega-3 fatty acids and risk of lung cancer.

This study employed IVW, MR-Egger, weighted median, simple mode, and weighted mode approaches to estimate the association between omega-3 fatty acids and risk of lung cancer. Results from IVW, MR-Egger, weighted median, and weighted mode approaches all showed that omega-3 fatty acids were casually associated with low risk of lung cancer. IVW, MR-Egger, and weighted median are commonly applied approaches in MR analyses [26]. Each approach has its own advantages and disadvantages in the consistency and test performance of causal effect estimation, and the performance of causal effect is also different due to unverifiable assumptions [27]. The effectiveness of the IVW method in finding causal effects is higher than that of weighted median method and MR-Egger analysis [28]. However, due to the strong assumptions that the IVW method relies on, the type I error rate of causal effect estimation and the bias of the estimated value of causal effect are caused by the IVW method [29]. The MR-Egger method is greatly affected by the inside hypothesis [30]. When the inside hypothesis is satisfied, the type I error rate of the causal effect estimation and the bias of the gene pleiotropy effect can be well controlled; once the inside hypothesis is violated, its test performance greatly affects [31]. For the weighted median method, when the inside assumption is violated, if there are not too many invalid instrumental variables, its performance is better than the other two methods [32]. There are two types of pleiotropy (horizontal pleiotropy as well as vertical pleiotropy) [33, 34]. Horizontal pleiotropy will occur if the second phenotype is in a distinct biological pathway [35]. Therefore, there might be distinct causal pathways from variation to outcomes and this could violate the IV3 assumption [36]. Vertical pleiotropy will occur if a variant shows direct correlations to exposure on the same biological pathway as well as another phenotype, which cannot result in a violation of the IV assumption and can provide a unique causal pathway from genetic variation to outcomes through exposure [37]. Horizontal pleiotropy can produce bias when SNPs presented associations with confounders via pathways that did not involve omega-3 fatty acids [38]. Nevertheless, our results from MR-Egger, weighted median, and weighted mode approaches with less effect on horizontal pleiotropy showed similarity to IVW estimates [39]. Furthermore, excluding SNPs that presented highly significant correlations to lung cancer causal factors possessed minimal effects on the estimates. Our Cochran's Q of IVM analysis showed that there was no heterogeneity among SNPs; moreover, MR-Egger regression analysis demonstrated that SNPs could have no-horizontal pleiotropy between omega-3 fatty acids and risk of lung cancer. When utilizing a single SNP as an IV, the point representative of the causal association effect was symmetric distribution, indicating that the cause was less likely to be influenced by potential bias.

Omega-3 fatty acid supplements have been studied for chemo-preventing human cancers, including lung cancer [40]. As immuno-nutrients, omega-3 fatty acids are often applied in nutritional treatment of cancer [41]. They exert a crucial role in cell signaling, cell structure, and cell membrane fluidity [42]. Furthermore, they mediate the resolution of inflammation, thereby exerting an anti-inflammation effect [43]. A meta-analysis showed that omega-3 fatty acid intake did not display a significant correlation to lung cancer [16]. However, a clinical study demonstrated that omega-3 fatty acid supplements are enabled to improve nutritional status and inhibit the systemic inflammatory response for lung cancer patients [15]. Differently, another retrospective study found that omega-3 fatty acids can reduce C-reactive protein and interleukin-6 levels for advanced NSCLC patients, but not affected nutritional status [44]. Our MR analyses demonstrated the casual relationship of omega-3 fatty acids with risk of lung cancer.

Compared with other studies, the advantages of this study are as follows: firstly, MR analyses can prevent reverse causality caused by inherent confounding factors in traditional observational studies; secondly, the study sample was larger, which could increase the statistical effect and result in a relatively more precise effect estimate. However, there are several limitations of this study: firstly, public data from UK Biobank and ILCCO were used, and the included study populations were mainly from European countries. Whether the conclusions of the study are applicable to other populations remains to be verified universally. Secondly, the study cohort of lung cancer patients cannot be directly obtained. Therefore, the subgroup analysis cannot be carried out. Thirdly, the potential biological mechanism between omega-3 fatty acids and risk of lung cancer is still not completely clear, and the MR method can only make a preliminary judgment on their causal relationship.

## 5. Conclusion

Collectively, our MR analyses offered strong evidence to demonstrate that omega-3 fatty acids exert a causal role in reducing the risk of lung cancer. Moreover, in-depth work is required for elucidating the underlying mechanisms that mediate the relationship of omega-3 fatty acids with lung cancer.

## Figures and Tables

**Figure 1:** Forest plot of single-nucleotide polymorphisms (SNPs) associated with omega-3 fatty acids and risk of lung cancer. Each black point indicates the log odds ratio (OR) for lung cancer per standard deviation (SD) increase in omega-3 fatty acids, generated utilizing each omega-3 fatty acids-associated SNP as an instrument. The horizontal line denotes 95% confidence intervals of the estimates. The red point shows the combined causal estimates utilizing all SNPs as an instrument based on MR-Egger and inverse-variance weighted (IVW) approaches.

**Figure 2:** Scatter plot of SNPs associated with omega-3 fatty acids and risk of lung cancer. The plot shows the SNP effects on omega-3 fatty acids (*x*-axis, SD units) as well as lung cancer (*y*-axis, log odds ratio (OR)) with 95% confidence intervals. The Mendelian randomization (MR) regression slopes of the lines represent the causal estimates using five approaches (inverse-variance weighted (IVW), MR-Egger, weighted median, simple mode, and weighted mode).

**Figure 3:** Funnel plot of causal associations between omega-3 fatty acids and risk of lung cancer.

**Table 1:** Detailed information of studies included and predictive strength of IVs in Mendelian randomization analyses (two-sided *α* = 0.05).

Exposures/outcomes	Consortium	Ethnicity	Sample sizes	nSNP
Omega-3 fatty acids	UK Biobank	European	114,999	12,321,875
Lung cancer	ILCCO	European	18,313	8,893,750

ILCCO: International Lung Cancer Consortium; SNP: single-nucleotide polymorphism; nSNP: number of SNPs.

**Table 2:** Harmonized dataset of univariate Mendelian randomization for the effect of omega-3 fatty acids on lung cancer.

SNP	EA exposure	Other allele exposure	EA outcome	Other allele outcome	Chromosome	Exposure			Outcome		
						*β*	SE	*p*	*β*	SE	*p*
rs10184054	G	C	G	C	2	-0.036	0.005	5.6*E* − 15	0.006	0.021	0.776
rs10455872	G	A	G	A	6	-0.063	0.008	2.8*E* − 17	-0.028	0.044	0.564
rs11242109	T	G	T	G	5	0.024	0.004	2.4*E* − 09	0.036	0.019	0.047
rs112875651	A	G	A	G	8	-0.087	0.004	3.5*E* − 98	0.007	0.019	0.702
rs1132899	C	T	C	T	19	0.027	0.004	8.6*E* − 11	-0.009	0.018	0.619
rs11563251	T	C	T	C	2	0.035	0.006	3.2*E* − 08	0.041	0.031	0.178
rs1167998	A	C	A	C	1	0.071	0.004	3.6*E* − 66	-0.036	0.020	0.061
rs11681659	T	C	T	C	2	-0.025	0.004	2*E* − 08	-5E-04	0.020	0.981
rs117143374	C	T	C	T	21	-0.037	0.006	2.2*E* − 10	0.059	0.028	0.028
rs117733303	G	A	G	A	6	-0.116	0.015	1.4*E* − 15	-0.138	0.057	0.048
rs12226389	C	T	C	T	11	-0.051	0.005	1.1*E* − 22	-0.045	0.026	0.099
rs1260326	C	T	C	T	2	-0.082	0.004	8.4*E* − 88	0.004	0.018	0.841
rs13424225	T	G	T	G	2	0.022	0.004	2.2*E* − 08	0.011	0.018	0.571
rs139974673	C	T	C	T	15	0.118	0.013	2.3*E* − 21	-0.1	0.047	0.068
rs143355652	T	C	T	C	11	-0.154	0.020	9.4*E* − 14	-0.047	0.084	0.628
rs1672811	C	T	C	T	16	0.025	0.005	3*E* − 08	-0.016	0.020	0.431
rs174564	G	A	G	A	11	-0.337	0.004	1*E* − 200	-0.061	0.018	0.002
rs1800978	G	C	G	C	9	-0.037	0.006	5.2*E* − 09	0.033	0.028	0.234
rs261290	C	T	C	T	15	-0.114	0.004	4*E* − 161	-0.005	0.019	0.778
rs3018731	G	A	G	A	11	-0.035	0.005	2*E* − 14	0.008	0.025	0.744
rs34663616	A	C	A	C	15	0.036	0.006	4.4*E* − 10	-0.044	0.028	0.143
rs35135293	T	C	T	C	2	-0.021	0.004	3.9*E* − 08	-0.005	0.018	0.773
rs4000713	A	G	A	G	7	-0.029	0.004	1*E* − 11	-0.019	0.019	0.349
rs58542926	T	C	T	C	19	-0.172	0.008	1*E* − 113	-0.038	0.033	0.288
rs6129624	A	G	A	G	20	-0.026	0.004	5.1*E* − 10	-0.023	0.019	0.243
rs62466318	T	C	T	C	7	-0.072	0.005	1.2*E* − 45	0.059	0.025	0.015
rs629301	T	G	T	G	1	0.038	0.005	1.3*E* − 14	0.02	0.021	0.359
rs633695	G	A	G	A	15	0.084	0.004	9.1*E* − 80	-0.013	0.019	0.526
rs6601924	C	T	C	T	10	0.035	0.006	8.5*E* − 10	0.006	0.025	0.829
rs6693447	G	T	G	T	1	0.023	0.004	4.8*E* − 09	0.041	0.019	0.033
rs673335	C	T	C	T	11	-0.067	0.006	1.1*E* − 34	0.024	0.024	0.325
rs6882345	A	G	A	G	5	0.029	0.004	1.9*E* − 13	-0.016	0.019	0.388
rs72789541	A	T	A	T	16	-0.081	0.004	5.6*E* − 75	-0.01	0.020	0.624
rs73109460	A	G	A	G	7	-0.035	0.006	9.2*E* − 10	0.024	0.031	0.447
rs737338	T	C	T	C	19	-0.073	0.011	3.5*E* − 11	-0.024	0.040	0.576
rs77960347	G	A	G	A	18	0.162	0.018	7.2*E* − 22	0.070	0.085	0.413
rs7819706	G	A	G	A	8	-0.040	0.006	1.8*E* − 10	3E-04	0.026	0.990
rs7924036	T	G	T	G	10	0.023	0.004	5.5*E* − 10	-0.005	0.018	0.778
rs7970695	A	G	A	G	12	-0.025	0.004	1.2*E* − 10	-0.013	0.019	0.472
rs9304381	T	C	T	C	18	0.053	0.005	5.2*E* − 24	-0.004	0.024	0.884
rs964184	C	G	C	G	11	-0.117	0.006	8.9*E* − 87	-0.037	0.026	0.155
rs9987289	G	A	G	A	8	0.057	0.007	3.2*E* − 16	-0.04	0.032	0.199

SNP: single-nucleotide polymorphism; SE: standard error; EA: effect allele; *β*: effect value.

**Table 3:** Associations of omega-3 fatty acids with lung cancer in Mendelian randomization analysis.

MR					Heterogeneity			Pleiotropy	
Methods	nSNP	Beta	OR (95% CI)	*p*	Method	Cochran's Q	*p*	Egger-intercept (95% CI)	*p*
IVW	42	-0.106	0.899 (0.817, 0.990)	0.03	IVW	69.8	0. 240	0.006 (-0.006, 0.018)	0.293
MR-Egger	42	-0.156	0.856 (0.750, 0.977)	0.026					
Weighted median	42	-0.175	0.899 (0.817, 0.990)	0.001					
Simple mode	42	-0.104	0.901 (-0.678, 1.199)	0.478					
Weighted mode	42	-0.152	0.859 (0.782, 0.944)	0.003					

MR: Mendelian randomization; SNP: single-nucleotide polymorphism; nSNP: number of SNPs; OR: odds ratio; CI: confidence interval; IVW: inverse variance weighted.

## Data Availability

The datasets analyzed during the current study are available from the corresponding author on reasonable request.

## Abbreviations

SCLC: Small-cell lung carcinoma
NSCLC: Non-SCLC
CT: Computed tomography
ALA: *α*-Linolenic acid
EPA: Eicosapentaenoic acid
DHA: Docosahexaenoic acid
MR: Mendelian randomization
SNPs: Single-nucleotide polymorphisms
IVs: Instrumental variables
GWAS: Genome-wide association study
ILCCO: International Lung Cancer Consortium
LD: Linkage disequilibrium
SEs: Standard errors
OR: Odds ratio
CI: Confidence intervals
IVW: Inverse variance weighted.
